RETRACTED

# Changes and Prognostic Value of lncRNA CASC9 in Patients with Advanced Colon Cancer after Chemotherapy

**DOI:** 10.1155/2021/1858974

**Published:** 2021-09-18

**Authors:** Yingwei Jiao, Qiang Liu, Hongbo Zhao, Xianzhen Hu, Jinlong Sun, Xiaohong Liu

**Affiliations:** ^1^Department of Proctology, Shaanxi Nuclear Industry 215 Hospital, Xianyang, Shaanxi 712000, China; ^2^Four Departments of General Surgery, Shaanxi Nuclear Industry 215 Hospital, Xianyang, Shaanxi 712000, China; ^3^Department of Traditional Chinese Medicine, Baoji Maternal and Child Health Care Hospital, Baoji, Shaanxi 721000, China

## Abstract

**Objective:**

Colon cancer (CC) shows a gradual increasing incidence in recent years, and chemotherapy is a frequently adopted treatment for patients with middle or advanced colon cancer (ACC), but it lacks prognostic markers after CC.

**Methods:**

The changes of lncRNA CASC9 in 58 patients with CC were determined using a real-time quantitative PCR (qRT-PCR) assay before and after chemotherapy, and the correlation of serum lncRNA CASC9 with efficacy of FOLFOX4 regimen (oxaliplatin + calcium folinate + fluorouracil) was analyzed. The patients were followed up to understand the association of lncRNA CASC9 with overall survival (OS) and progression-free survival (PFS).

**Results:**

Patients with CC showed notably higher lncRNA CASC9 expression than controls, and lncRNA CASC9 presented an association with the clinical stage of the patients. In addition, lncRNA CASC9 demonstrated a clinical value in predicting efficacy on patients and acted as one independent prognostic factor for PFS in patients with ACC.

**Conclusions:**

With increased expression of serum lncRNA CASC9, patients with ACC suffered an unfavorable chemotherapy effect. In addition, serum lncRNA CASC9 is a promising sensitive indicator for prediction of ACC and is related to the clinical efficacy and prognosis of patients.

## 1. Introduction

As a frequently seen cancer worldwide, colon cancer (CC) ranks the third in malignant tumor and the second in the causes of cancer-associated deaths in recent years [1]. Despite the advancement in treatment against CC over the past few decades, the treatment results still depend to some extent on the unique molecular characteristics of tumors and patients [2, 3]. At the current stage, novel drugs against CC emerge constantly [4, 5]. However, the survival rate of patients with cancer is still unsatisfactory. In the past decade, the new biotherapy of monoclonal antibodies has demonstrated a powerful ability to improve the clinical prognosis of patients [6], but there are still a large proportion of patients who do not benefit from the treatment [7]. In addition, prognostic indicators of CC are wanting in clinical practice. One earlier study has revealed the predictive value of biological markers for the prognosis of patients [8].

RETRACTED

Long-chain noncoding RNA (lncRNA) is a transcription factor longer than 200 nucleotides and is deemed as a waste product produced by the metabolism due to the absence of protein coding ability [9]. Additionally, lncRNA has exhibited regulation functions in many mechanisms, including epigenetic modification, transcriptional regulation, and posttranscriptional modification [10], and has also showed its potential to be a diagnostic marker of cancer [11]. lncRNA cancer susceptibility candidate 9 (CASC9) is an lncRNA situated at human 8q21.13 chromosome. Earlier studies have revealed its expression in cases with liver cancer and those with bladder cancer and its association with tumor prognosis [12, 13]. Moreover, one recent study has found its expression in cases with colorectal cancer (CRC) [14], which suggests that lncRNA CASC9 is probably a potential biomarker of CRC.

In this study, we primarily quantified lncRNA CASC9 in patients with advanced colon cancer (ACC) and analyzed its prognostic value for such patients, with the goal of providing promising prognostic markers for CC in clinical practice.

## 2. Methods and Materials

### 2.1. Clinical Data

Totally, 58 patients with ACC admitted to our hospital between January 2017 and January 2019 were enrolled, including 38 males and 20 females, aged 45–71 years, with a median age of 62 years, and 30 patients with early CC treated in our hospital over the same time span were also enrolled, including 20 males and 10 females, aged 42–75 years, with a median age of 57 years. In addition, 30 healthy individuals who underwent physical examination in our hospital over the same time span were enrolled as controls, including 18 males and 12 females, aged 50–71 years, with a median age of 62 years. These participants were not greatly different in age and gender (both *P* > 0.05), and they all gave their signatures on informed consent forms after being apprised of the study. In addition, the study was performed with approval from the ethics committee of our hospital and was in agreement with the Declaration of Helsinki [15].

### 2.2. Inclusion and Exclusion Criteria

The inclusion criteria: patients confirmed with CC by imaging and pathological diagnosis, patients with CC at stage I or II (patients with early CC), patients with ACC at stage III or IV (patients with ACC), patients who had not experienced targeted therapy (surgery, radiotherapy, chemotherapy, and targeted therapy) before the study, and those with ACC who were expected to live longer than 3 months.

RETRACTED

The exclusion criteria: patients with other comorbid tumors, patients intolerant to drugs used in this study, and those reluctant to cooperate with follow-up.

### 2.3. Therapeutic Regimen

This study was primarily to probe into lncRNA CASC9 in the serum of patients with ACC before and after therapy, so the therapeutic regimen for patients with early CC was not described. Patients with middle or advanced CC were treated with FOLFOX4 regimen (oxaliplatin + calcium folinate + fluorouracil). Specifically, the patients were given 85 mg/m^2^ oxaliplatin for 2 h via intravenous drip on the first day, given 200 mg/m^2^ calcium folinate for 2 h via intravenous drip on the first day and second day, and also given 400 mg/m^2^ fluorouracil via intravenous injection, followed by continuous intravenous infusion of 600 mg/m^2^ fluorouracil via a micropump for 22 h on the first day and second day. A whole treatment cycle consisted of 14 days, and all patients must receive such chemotherapy for at least 3 cycles.

### 2.4. qRT-PCR Assay

Peripheral blood was sampled from each participant, and the serum was centrifugally obtained, followed by extraction of RNA in the serum with a TRIzol reagent (Invitrogen). Then, the RNA was treated by reverse transcription via a EasyScript® One-Step gDNA Removal and cDNA Synthesis SuperMix (TransGen, Beijing, China) and placed on a biological system 7500 (ABI, USA) for RCR amplification via the SYBR Premix Ex Taq II (Takara, Dalian, China) under 25 *μ*L total volume with SYBR Premix Ex Taq II (2X) (12.5 *μ*L), upstream primer (1 *μ*L), downstream primer (1 *μ*L), DNA template (2 *μ*L), and dH_2_O (8.5 *μ*L) through predenaturation (95°C, 10 s), followed by 40 cycles of denaturation (95°C, 5 s) and annealing extension (60°C, 30 s). Qualification was achieved according to 2^−ΔΔ*Ct*^ (internal reference of lncRNA CASC9: GAPDH) [16]. The upstream and downstream sequences of lncRNA CASC9 are 5'-TTGGTCAGCCACATTCATGGT-3' and 5'-AGTGCCAATGACTCTCCAGC-3'; the upstream and downstream sequences of GAPDH are 5'-GGGAGCCAAAAGGGTCATCA-3' and 5'-TGATGGCATGGACTGTGGTC-3'.

### 2.5. Outcome Measures

Primary outcome measures: serum lncRNA CASC9 in patients with CC was quantified, and its expression in these patients at different stages was also analyzed. After detecting the expression of lncRNA CASC9, the median of 2.38 was used as the standard for the expression of lncRNA CASC9. In addition, Cox regression analysis was carried out to understand factors affecting progression-free survival (PFS) and overall survival (OS) of patients with ACC.

Secondary outcome measures: the association of lncRNA CASC9 expression with clinical efficacy of chemotherapy in patients with ACC was analyzed, and the efficacy was evaluated according to the Response Evaluation Criteria in Solid Tumors (RECIST) [17].

RETRACTED

### 2.6. Statistical Analyses

This study adopted SPSS20.0 for statistical analyses of obtained data. Enumeration data (presented by %) were analyzed via the chi-square test and presented by 2, and ranked data were analyzed via the Mann–Whitney test and presented by Z. Additionally, the K-M survival curve was adopted for visualizing the OS of patients and the log-rank test for analyzing independent factors impacting the prognosis of patients. Receiver operating characteristic (ROC) curve was adopted for the predictive value analysis of lncRNA CASC9 for survival of and clinical efficacy on patients with ACC. Moreover, Spearman correlation was used for association analysis between lncRNA CASC9 and clinical efficacy. *P* < 0.05 denotes a remarkable difference.

## 3. Results

### 3.1. LncRNA CASC9 Expression in Patients with CC

We first analyzed lncRNA CASC9 expression in cases with colon adenocarcinoma according to the TCGA database by GEPIA2 online web and found notably higher lncRNA CASC9 in cases with colon adenocarcinoma than that in control specimens (Figure 1(a), *P* < 0.001). Then, we carried out a qRT-PCR assay and also found higher lncRNA CASC9 in cases with CC and its remarkably higher expression than that in controls (Figure 1(b), *P* < 0.001).

### 3.2. Value of lncRNA CASC9 Expression for CC Staging

With the aim of more deeply understanding lncRNA CASC9 in patients with CC, we grouped the patients according to their cancer stage and then analyzed its expression in patients with different clinical stages. Analysis showed that patients with higher lncRNA CASC9 had notably higher CC stage (Figure 2, *P* < 0.001).

### 3.3. Correlation of lncRNA CASC9 Expression with Clinical Efficacy of Chemotherapy on Patients with ACC

Through the above analysis, we discovered association of lncRNA CASC9 with clinical CC stage of patients. We further probed into the correlation of lncRNA CASC9 with clinical efficacy of chemotherapy on patients with ACC. The results showed 5 cases of complete remission (CR), 20 cases of partial response (PR), 24 cases of stable disease (SD), and 9 cases of progressive disease (PD) after chemotherapy. According to analysis, lncRNA CASC9 in the serum of patients showed lower relative expression after chemotherapy (Figure 3(a), *P* < 0.001), and further analysis revealed its positive correlation with clinical efficacy in patients (Figure 3(b), *P* < 0.001). In addition, for understanding the value of lncRNA CASC9 in forecasting the clinical efficacy on patients with ACC, we assigned patients with CR, PR, or SD into a nonprogressive group and those with PD into a progressive group. As a result, the former presented lower lncRNA CASC9 expression than the latter (Figure 3(c), *P* < 0.001). Moreover, the ROC curve-based analysis revealed that lncRNA CASC9 expression was of clinical significance in forecasting clinical efficacy on patients (Figure 3(d), *P* < 0.001).

RETRACTED

### 3.4. Cox Regression Analysis

We also carried out a Cox regression analysis to understand influencing factors of PFS and OS. The univariate analysis revealed that clinical stage, lymph node metastasis (LNM), and lncRNA CASC9 were all prognostic factors of PFS in patients with ACC, and the latter two were prognostic factors of OS in them (Table 1, all *P* < 0.05). The above indices were included for the multivariate Cox regression analysis, which revealed that the three were all independent prognostic factors of PFS in patients with ACC, and clinical stage and LNM were independent prognostic factors of OS in them (Table 2, *P* < 0.05).

### 3.5. Survival Curve about Independent Risk Factors of PFS and OS

Exploring the survival curves of independent risk factors for PFS and OS, it was found that patients with clinical staging (IV), number of lymph node metastases (≥12), and lncRNA CASC9 (≥2.38) have shorter PFS. Patients with clinical staging (IV) and number of lymph node metastases (≥12) have shorter OS (Figure 4, *P* < 0.05).

## 4. Discussion

ACC has always been a tricky problem in clinical practice [18]. At the present stage, patients with ACC are primarily treated by chemotherapy that commonly involves 3 categories of drugs, namely, 5-FU and its derivatives, the third-generation platinum drugs, and topoisomerase I inhibitors [19]. However, the individual differences and severe side effects in patients limit the clinical application of chemotherapeutic drugs to a certain extent and even give rise to chemotherapy failure. According to one recent study, the changes of biomarkers can help predict and evaluate the prognosis of patients [20].

lncRNA is a potential biomarker that has captured much attention over the past few years [21]. One earlier study has revealed the involvement of lncRNA in the development of various cancers and has also pointed out that lncRNA CASC9 is a novel tumor susceptibility gene [22]. In addition, in one study [23], lncRNA CASC9 accelerated the metastasis of esophageal squamous cell carcinoma through upregulating LAMC2 by interaction with CREB binding protein. However, reports about lncRNA CASC9 in CC are scarce, and whether it can be a prognostic indicator of CC requires further study. Our study first analyzed lncRNA CASC9 expression in cases with colon adenocarcinoma according to the TCGA database by GEPIA2 online web and found notably high lncRNA CASC9 expression in cases with colon adenocarcinoma and also verifies the high expression through a qRT-PCR assay. Furthermore, we also found patients at a higher CC stage presented notably higher lncRNA CASC9 expression, which suggested the involvement of lncRNA CASC9 in the development of CC.

RETRACTED

With the aim of more deeply understanding the value of lncRNA CASC9 in ACC, we evaluated its expression in cases with the disease before and after therapy. Our analysis revealed its positive correlation with clinical efficacy on patients and its increase with the deterioration of the efficacy. In addition, we found lncRNA CASC9 in patients with progressive disease increased greatly and demonstrated a potential predictive value. These results imply the relatively high clinical significance of lncRNA CASC9 in patients with ACC. One earlier study has revealed the high expression of lncRNA CASC9 in cases with gastric cancer (GC) and even higher expression of it in BGC823/DR and SGC7901/DR cells resistant to paclitaxel or adriamycin, but knocking down lncRNA CASC9 in the drug-resistant cell stains restored the chemical sensitivity of GC cells to paclitaxel and adriamycin in this study [24]. Moreover, one study by Jiang et al. [25] has found higher lncRNA CASC9 in epirubicin-resistant breast cancer cells (BCC**s)** than that in nondrug-resistant BCCs and has also restored the chemical sensitivity of BCCs to epirubicin by knocking down lncRNA CASC9 [25]. These results indicate the involvement of lncRNA CASC9 in the development of CC. In our study, patients with high lncRNA CASC9 expression acquired unfavorable clinical efficacy after chemotherapy, which might explain the fact that the sensitivity of tumor cells to chemotherapeutic drugs decreased due to the excessive expression of lncRNA CASC9, and finally, the chemotherapy was ineffective or even a failure. Finally, we analyzed the prognostic factors of PFS and OS in patients with ACC. Our analysis showed that lncRNA CASC9 was an independent prognostic factor impacting PFS in patients with ACC. These results denote that lncRNA CASC9 is a promising biomarker for prognosis observation of patients with ACC.

Through the above research, we have confirmed the clinical significance of lncRNA CASC9 in patients with ACC. However, this study still has some limitations. First, although we have confirmed the clinical significance of lncRNA CASC9 in patients with ACC, we have not more deeply analyzed the mechanism of drug resistance. Second, the sample of this study is relatively simple, and we have not tested the tumor tissues of patients. However, some studies have revealed that besides serum, lncRNA expression in exosomes of peripheral blood/tumor tissues and peripheral blood mononuclear cells of patients with tumors is also of high diagnostic and prognostic value [26, 27]. Finally, the clinical sample size of this study is small, and the patients have not been followed up for a long time. Therefore, we hope to address our research limitations and improve our conclusions in future research.

RETRACTED

To sum up, with increased expression of serum lncRNA CASC9, patients with ACC suffered an unfavorable chemotherapy effect. In addition, serum lncRNA CASC9 is a promising sensitive indicator for efficacy prediction of chemotherapeutic drugs.

## Figures and Tables

**Figure 1:** LncRNA CASC9 expression in patients with CC. (a) LncRNA CASC9 expression in patients with CC according to GEPIA2 online analysis. (b) Serum lncRNA CASC9 expression in cases with CC according to the qRT-PCR assay. ^*∗*^*P* < 0.05. ^*∗∗∗*^*P* < 0.001.

**Figure 2:** Serum lncRNA CASC9 in patients with different stages according to the qRT-PCR assay. ^*∗*^*P* < 0.05. ^*∗∗*^*P* < 0.01. ^*∗∗∗*^*P* < 0.001.

**Figure 3:** Correlation of lncRNA CASC9 with clinical efficacy of chemotherapy on patients with ACC. (a) Changes of serum lncRNA CASC9 expression in patients with ACC before and after therapy. (b) Correlation analysis between lncRNA CASC9 expression and clinical efficacy before therapy. (c) LncRNA CASC9 expression in the nonprogressive group and the progressive group. (d) Area under the ROC curve of lncRNA CASC9 expression in predicting the progress of patients. ^*∗∗*^*P* < 0.01. ^*∗∗∗*^*P* < 0.001.

**Figure 4:** Survival curve about independent risk factors of PFS and OS. (a) Survival curve of different clinical stages in PFS. (b) Survival curve of LNM number in PFS. (c) Survival curve of lncRNA CASC9 in PFS. (d) Survival curve of different clinical stages in OS. (e) Survival curve of LNM number in OS.

**Table 1:** Univariate analysis.

Factors	Single factors of PFS			Single factor of OS		
	*P* value	HR value	95% CI	*P* value	HR value	95% CI

Age (≥60 years vs. <60 years)	0.437	1.231	0.729–2.080	0.736	1.096	0.644–1.864
Sex (male vs. female)	0.576	0.855	0.494–1.481	0.871	0.956	0.552–1.656
Clinical staging (III vs. IV)	0.497	0.834	0.495–1.407	0.006	2.272	1.272–4.055
Number of lymph node metastases (≥12 vs. <12)	0.674	0.895	0.533–1.501	0.012	0.490	0.280–0.858
Location of lesion (left colon vs. right colon)	0.185	1.424	0.845–2.401	0.657	1.128	0.663–1.920
lncRNA CASC9 (≥2.38 vs. <2.38)	0.014	2.079	1.160–3.727	0.941	1.022	0.571–1.829

**Table 2:** Multivariate analysis.

Factors	Single factors of PFS			Single factor of OS		
	*P* value	HR value	95% CI	*P* value	HR value	95 CI%

Age (≥60 years vs. <60 years)	0.296	0.742	0.424–1.298	0.959	1.014	0.589–1.747
Sex (male vs. female)	0.867	0.952	0.538–1.686	0.803	0.924	0.497–1.719
Clinical staging (III vs. IV)	0.004	2.615	1.367–5.001	0.002	2.555	1.393–4.687
Number of lymph node metastases (≥12 vs. <12)	0.001	0.331	0.172–0.638	0.008	0.456	0.256–0.812
Location of lesion (left colon vs. right colon)	0.207	1.424	0.822–2.466	0.459	1.23	0.711–2.127
lncRNA CASC9 (≥2.38 vs. <2.38)	<0.001	3.716	1.879–7.352	0.513	1.25	0.64–2.441

RETRACTED

## Data Availability

The data used and/or analyzed in this study are available from the corresponding author upon request.
